This article has been retracted.

# Downregulated Expression of miRNA-130a-5p Aggravates Hepatoma Progression via Targeting PTP4A2

**DOI:** 10.1155/2021/4439505

**Published:** 2021-12-28

**Authors:** Longqing Shi, Fengbo Wang, Yue Zhang, Yue Yang, Zheng Qu, Donglin Sun

**Affiliations:** ^1^Department of Hepatobiliary and Pancreatic Surgery, The Third Affiliated Hospital of Soochow University, Jiangsu, China; ^2^Department of Neurosurgery, Xinyi People's Hospital, Jiangsu, China

## Abstract

**Background:**

Hepatoma is a leading cause of death worldwide, with high metastasis and recurrence rates. The aberrant expression of miRNA-130a-5p is involved in the development and progression of various cancers. However, there are no studies investigating the role of miRNA-130a-5p in hepatoma. The present study is aimed at clarifying the functional role of miRNA-130a-5p in hepatoma progression.

**Methods:**

The expression levels of miRNA-130a-5p in hepatoma tissues and cell lines were detected by qRT-PCR assays. Bioinformatic analysis, gain-/loss-of-function experiments, and luciferase activity assays were conducted to verify whether miRNA-130a-5p is targeted by protein tyrosine phosphatase 4A2 (PTP4A2). The functions of miRNA-130a-5p and PTP4A2 in hepatoma were determined by cell proliferation assays.

**Results:**

The expression of miRNA-130a-5p was downregulated in hepatoma tissues and was related to poor prognosis. However, the expression level of PTP4A2 was contradictory to that of miRNA-130a-5p, and PTP4A2 upregulation could aggravate hepatoma progression. The ectopic overexpression of PTP4A2 promoted hepatoma cell proliferation in vitro, which could be reversed by miRNA-130a-5p.

**Conclusions:**

Our study implies that miRNA-130a-5p, which is downregulated in hepatoma tissues, can suppress hepatoma cell proliferation via targeting PTP4A2.

## 1. Introduction

Hepatoma is a leading cause of cancer-related death, which accounts for >90% of patients with liver cancer [1]. The majority of hepatoma patients are diagnosed at advanced stages, thus leading to a high mortality rate [2]. Over the past decades, considerable progresses have been made in the diagnosis and treatment of hepatoma, but the results are not quite satisfactory [3]. Growing evidence demonstrates that molecular targeted therapy holds a great promise for treating hepatoma patients [4], but the underlying mechanisms of hepatoma progression await further studies.

microRNA (miRNA), as a research hotspot in recent decades, has been reported to play a significant role in cancer progression [5]. For instance, miRNA-106b-5p is an oncogene involved in breast cancer cell metastasis [6]. Tian et al. [7] found that miRNA-21 and miRNA-10b can act as tumor promoters in hepatoma. Moreover, miRNA-155 has been acknowledged in cancer drug resistance and as a target for miRNA-based therapy. Several reports have demonstrated that miRNA-130a-5p is aberrantly expressed in various cancers, including lung cancer [8], gastric carcinoma [9], and renal carcinoma [10]. Besides, miRNA-130a-5p can also regulate chemosensitivity, proliferation, and metastasis in tumor cells. However, the precise role of miRNA-130a-5p in hepatoma is still unknown.

The protein tyrosine phosphatase 4A (PTP4A) family, or known as phosphatase of regenerating liver (PRL), is consisted of PTP4A1-3/PRL1-3, which has been implicated in tumor progression and oncogenesis [11]. In human breast cancer, PTP4A2 predicts the overall and disease-free survival of cancer patients [12]. PTP4A2 is also responsible for governing the transition of cell cycle from the G1 to the S phase [13].

Herein, we found that miRNA-130a-5p was downregulated in hepatoma tissues and cell lines, leading to a poor prognosis in hepatoma patients. miRNA-130a-5p could act as an inhibitor of hepatoma by decreasing cell proliferation. In addition, miRNA-130a-5p was directly targeted by PTP4A2 in hepatoma cells. PTP4A2 could reverse the inhibitory effect of miRNA-130a-5p on hepatoma cell proliferation. Altogether, our study reveals that miRNA-130a-5p plays a crucial role in hepatoma progression via targeting PTP4A2.

## 2. Materials and Methods

### 2.1. Cell Lines and Culture

The cell lines HepG2, Hep3B, HCCLM3, Huh-7, MHCC-97L, MHCC-97H, and SMMC-7721 were cultured in DMEM medium (Gibco, 11995-065, MD, USA) containing 10% fetal bovine serum (FBS, Gibco) and 100 U/mL penicillin-streptomycin mixture (Gibco) in a 5% CO_2_ incubator at 37°C. The cells were harvested at the indicated time points. RNA and protein were extracted for independent experiments.

### 2.2. Tissue Samples

Tissue samples were obtained from The Third Affiliated Hospital of Soochow University, including hepatoma tissue and matched adjacent tissue samples from patients treated with surgery alone. All specimens were stored in frozen or formalin preservation solution. The study protocol was approved by the Ethics Committee. Written informed consent was provided by all patients for the use of their tissue specimens.

### 2.3. cDNA Synthesis and qRT-PCR Assays

Total RNA was extracted from hepatoma tissues and cells using the TRIzol Reagent (Invitrogen, USA). RNA quantification was performed using a NanoDrop2000c. PrimeScript RT Reagent kit (TaKaRa, RR047A) was used to reverse-transcribe total RNA into cDNA for qRT-PCR analysis. Then, quantitative real-time PCR assays were conducted on an ABI7500 system according to the protocols obtained from the manufacturers. The primer sequences used for qRT-PCR were as follows: miRNA-130a-5p: F: 5′-ACACTCCAGCTGGGGCTCTTT TCACATTGT-3′, R: 5′-CTCAACTGGT GTCGTGGAGTCGGCAATTCAGTTGAGAGTAGCAC-3′; GAPDH: F: 5′-TGTTC GTCATGG GTGT GAAC, R: 5′-ATGGCATGGACTGTGGTCAT3′; PTP4A2: F: 5′-AGATCTCCTATGAGAA CATGC-3′, R: 5′-TTGGAATTGAAC GCTCCC-3′.

### 2.4. Transient and Stable Cell Transfection

All oligonucleotides, including LV-miRNA-130a-5p, LV-PTP4A2, shPTP4A2, and small interfering RNA (siRNA) targeting miRNA-130a-5p and their corresponding controls, were commercially supplied by Gene-Pharma (Shanghai, China). The lentiviral vector was transfected into HCC-LM3 and Hep3B according to the kit's protocol. The siRNA sequence targeting miRNA-130a-5p was transfected with Lipofectamine 3000 reagent.

### 2.5. CCK-8 Assay

The stably transfected Hep3B and HCC-LM3 cells were grown in 96-well plates (1 × 10^3^ cells/well). Then, a 10 *μ*L volume of CCK-8 solution (Dojindo, Tokyo, Japan) was added to all wells at 24, 48, and 72 h, followed by incubation at 37°C for another 2 h. Subsequently, the absorbance was recorded using a microplate reader (450 nm; Thermo Scientific).

### 2.6. Western Blotting

Total protein was isolated with RIPA lysis buffer (Thermo Scientific) and PMSF (Beyotime) according to the manufacturer's protocols. The protein samples were added to SDS-PAGE gels, followed by electrophoresis. Subsequently, the protein samples were transferred onto PVDF membranes. After blocking with Quick-Block buffer (Beyotime) for 10 min, overnight incubation with the antibodies against PTP4A2/PRL2 (ab181776; Abcam) and GADPH (ab109118; Abcam) was performed at 4°C. After washing in TBST three times within 45 min, the secondary antibody was added and incubated at room temperature for 2 h. Lastly, the protein blots were examined using an ECL system (Sigma). The grey intensity of each protein band was quantified with ImageJ software.

### 2.7. Luciferase Reporter Assay

Hepatoma cells at 75% confluence were transfected with plasmids and miRNA-130a-5p inhibitors or miRNA-130a-5p mimics. Dual-Luciferase Reporter Assay System (Promega, WI, USA) was utilized to evaluate the luciferase activities after normalization to Renilla activity. First, Double Glo® Luciferase buffer was added to Dual-Glo® in a luciferase substrate bottle. Next, the substrate was completely dissolved to form Dual-Glo® Luciferase reagent, followed by subpackaging and storage at -70°C. Then, 250 *μ*l of medium was removed from each well in the 24-well plates, and the same amount of Dual-Glo was added into the remaining volume of ® Luciferase reagent and incubated at room temperature for 10 min until the cells were fully lysed. After mixing and transferring to a sterile 1.5 mL EP tube, Dual-Glo was prepared according to the required amount of freshly prepared ® Stop & Glo® Reagent. Later, 100 *μ*l of cell lysate was placed into the LockWell Maximorp detection plate, and the firefly fluorescence was detected using a microplate reader. In this step, the cells were treated with a Dual-Glo® Luciferase reagent and then incubated for 10-120 min. After detecting the firefly luminescence, 50 *μ*l of Dual-Glo® and Stop & Glo® Reagent was added into each well and incubated at room temperature. The detection of Renilla luminescence was completed within 10-120 min, and the detection time point was far from Dual-Glo® Stop & Glo®. The time point of reagent addition shall be the same as the time point of fire luminescence detection. Dual-Glo® Luciferase reagent was added at the same time point.

### 2.8. Colony Formation Assay

The cells (500 cells/well) were grown in 6-well plates and subjected to the evaluation of colony-forming ability. Colonies were observed every day for up to 10 days. Then, the medium was removed, followed by rinsing with PBS three times. After fixing in ethyl alcohol for 30 s, 1% crystal violet staining was conducted for 15 min. All colonies were manually counted.

### 2.9. Statistical Analyses

All values are shown as mean ± SD (standard deviation). Variations among the control and treatment groups were evaluated with Student's *t*-test. The *χ*^2^ test was employed to assess the relationships between miRNA-130a-5p expression and clinicopathological characteristics. The *P* values (^∗^*P* < 0.05; ^∗∗^*P* < 0.01; ^∗∗∗^*P* < 0.001) denote different levels of statistical significance. The correlation between the control and treatment groups, as well as the significance of the regression, was assessed by Pearson's correlation coefficients.

## 3. Results

### 3.1. Downregulated Expression of miRNA-130a-5p in Hepatoma Tissues and Cell Lines

To determine whether miRNA-130a-5p is involved in the progression of hepatoma, qRT-PCR was conducted on 40 pairs of hepatoma tissues and adjacent peritumoral tissues. The expression of miRNA-130a-5p was downregulated in hepatoma tissue compared with adjacent nontumor tissue (Figure 1(a)). The results were further confirmed using a bioinformatic tool (starBase) (Figure 1(b)). In addition, the expression of miRNA-130a-5p was detected in hepatoma cell lines. Compared with that in LO2 cells, miRNA-130a-5p was significantly decreased in HepG2, Hep3B, HCC-LM3, Huh-7, MHCC-97L, MHCC-97H, and SMMC-7721 cells (Figure 1(c)). To assess the correlations between miRNA-130a-5p and clinical data, hepatoma patients were categorized to high- and low-expression groups.

### 3.2. Correlation Analysis between Clinical Characteristics and miRNA-130a-5p in Patients with Hepatoma

MiRNAs have been proven to be effective and safe for predicting the prognostic outcomes of various diseases, including cancers [14]. The prognosis-related indicators of hepatoma patients include patient age, tumor characteristics, and AFP [15]. As demonstrated in Table 1, the expression level of miRNA-130a-5p was markedly correlated with tumor size (*P* = 0.004), TNM stage (*P* = 0.011), and Edmondson grade (*P* = 0.024), but did not correlate with age, gender, or AFP levels. These data indicate that miRNA-130a-5p can regulate the growth and differentiation of hepatoma.

### 3.3. Ectopic Overexpression of miRNA-130a-5p Inhibits Hepatoma Cell Proliferation

To assess the potential role of miRNA-130a-5p in hepatoma cell progression, HCC-LM3 and Hep3B cells were transfected with lentivirus vector micro-RNA-130a-5p (LV-miRNA-130a-5p) and miRNA-130a-5p siRNA, respectively. QRT-PCR was conducted to verify the transfection efficiencies. The expression levels of miRNA-130a-5p were upregulated and downregulated in HCC-LM3 cells transfected with LV-miRNA-130a-5p and Hep3B cells transfected with si-miRNA-130a-5p, respectively, compared to the negative control group (Figures 2(a) and 2(b)). The results of CCK-8 assay indicated that si-miRNA-130a-5p Hep3B cells grew more rapidly than the control cells (Figure 2(d)). At the same time, the miRNA-130a-5p overexpression decreased the proliferation rate of LM3 cells (Figure 2(c)). Besides, colony formation assays revealed that the miRNA-130a-5p overexpression in LM3 cells had antiproliferative activities (Figures 2(e)–2(h)). Therefore, the ectopic overexpression of miRNA-130a-5p remarkably attenuated hepatoma cell growth in vitro.

### 3.4. PTP4A2 Is Upregulated in Hepatoma Tissues and Related to Poor Survival

As miRNA-130a-5p could inhibit cell proliferation, bioinformatic databases (starBase, miRWalk, miRDB and Diana) were used to estimate potential downstream targets of miRNA-130a-5p (Figure 3(a)). Among them, PTP4A2 has attracted our attention since it plays crucial roles in modulating cell proliferation and cell cycle progression. The expression of PTP4A2 was analyzed based on TCGA datasets and 40 pairs of hepatoma tissues and corresponding adjacent tissues via qRT-PCR assays (Figures 3(b) and 3(d)). Compared with that in healthy tissues, the PTP4A2 expression was remarkably upregulated in hepatoma tissues (Figure 3(d)) but negatively related to the miRNA-130a-5p expression (Figure 3(c)). Kaplan-Meier curves showed that the PTP4A2 overexpression from TCGA was markedly associated with shorter survival in hepatoma patients (Figure 3(e)). Furthermore, miRNA-130a-5p negatively modulated the luciferase activity of wild-type PTP4A2-3' UTR compared with that of mutant-type (Figures 3(f) and 3(g)). QRT-PCR results showed that miRNA-130a-5p inhibitors upregulated the expression of PTP4A2 in Hep3B cells, while that of PTP4A2 in LM3 cells was downregulated by LV-miRNA-130a-5p (*P* < 0.001, *P* < 0.01, respectively; Figures 3(h) and 3(i)). Altogether, these data indicate that miRNA-130a-5p is directly targeted by PTP4A2.

### 3.5. PTP4A2 Overexpression Reverses the Effect of miRNA-130a-5p

To evaluate whether PTP4A2 can reverse the effect of miRNA-130a-5p on hepatoma cells, rescue experiments were performed via cotransfection assays. LM3 cells were transfected with PTP4A2 shRNA, miRNA-130a-5p inhibitors, and the respective controls in different combinations. Meanwhile, LV-PTP4A2, LV-miRNA-130a-5p, and the corresponding controls were transfected into Hep3B cells in different combinations. miRNA-130a-5p inhibitors upregulated the PTP4A2 expression in Hep3B cells (Figure 4(a)), while PTP4A2 shRNA attenuated the inductive effects of miRNA-130a-5p inhibitors on the PTP4A2 expression (Figure 4(a)). Moreover, LV-PTP4A2 partly enhanced the inductive effects of miRNA-130a-5p mimics on the PTP4A2 expression (Figure 4(b)). In addition, PTP4A2 shRNA partly diminished the effects of miRNA-130a-5p inhibitors on Hep3B proliferation (Figures 4(c) and 4(e)), while LV-PTP4A2 partly reversed the inhibitory effect of LV-miRNA-130a-5p on LM3 cell proliferation (Figures 4(d) and 4(f)). Collectively, our data implies that PTP4A2 can act as a key regulator of miRNA-130a-5p in hepatoma cells.

## 4. Discussion

miRNAs, a type of small regulatory RNAs, are commonly found in animals, plants, and other living organisms [16, 17]. miRNA dysregulation has been shown to be associated with hepatoma progression by modulating tumor cell growth and metastasis [18]. Therefore, it is necessary to develop an effective molecular therapy for hepatoma patients.

miRNA-130a-5p is a tumor suppressor gene and an endogenous molecular regulator associated with various human diseases. Runx2, a target transcription factor of miRNA-130a-5p, interacts with STK32a and regulates the miRNA-130a-5p expression. It also inhibits the migration, invasion, epithelial-mesenchymal transition (EMT), and viability of cancer cells, while promoting the apoptosis of non-small-cell lung cancer cells [19]. In gastric cancer, miRNA-130a-5p can inhibit the activation of Wnt/*β*-catenin pathway by targeting CB1R, bind to CCL22 targets, and negatively regulate CCL22 protein expression levels, thereby exerting antitumor effects and inhibiting gastric cancer progression [20]. It has also been reported that HOTAIR interacts with miRNA-130a-5p to regulate the ZEB1 expression, thus affecting the invasiveness and progression of esophageal squamous cell carcinoma, which provides a new therapeutic target for the early diagnosis and treatment of this disease [21].

However, the precise role of miRNA-130a-5p in hepatoma is still unclarified. In this work, the expression levels of miRNA-130a-5p in 40 hepatoma patients were detected, and it was noted that miRNA-130a-5p was remarkably downregulated in hepatoma tissues. To verify the results, we sought evidence from GEPIA tools. Consistently, we observed that the expression of miRNA-130a-5p was relatively lower in hepatoma tissues and hepatoma cell lines. In addition, the miRNA-130a-5p expression was significantly associated with tumor size, Edmondson grade, and TNM stage. These data indicate that miRNA-130a-5p can serve as a tumor inhibitor and prognostic marker for hepatoma. Furthermore, our findings demonstrate that miRNA-130a-5p may act as an inhibitor of hepatoma by decreasing the proliferation rates of tumor cells.

Previous research has suggested that miRNA exerts its influence by binding to the 3′-UTR of downstream targets [22]. In this study, the potential targets of miRNA-130a-5p were estimated using several bioinformatic tools. PTP4A2, which was predicted in common by all tools, had become our main focus. PTP4A2 belongs to the protein tyrosine phosphatase (PTP) gene family and is one of the most diverse in the mammalian genome, comprising 107 PTP genes [23]. PTP4A2 can dephosphorylate phosphatase and tensin homolog deleted on chromosome ten (PTEN) at y336, leading to partial loss of function of PTEN and ultimately tumorigenesis [24].

Previous studies have shown that PTP4A2 is a tumor promoter in different cancers. Its prognostic significance was assessed using the GEO database, and the results demonstrated that the PTP4A2 expression was correlated with survival time. Other studies have also found that PTP4A2 is significantly elevated in breast tumors and metastatic lymph nodes. The overexpression of PTP4A2 may promote breast cancer development through ERK pathway, leading to a rapid mammary tumor formation in breast cancer mice. Inhibition of PTP4A2 protein complex formation reduces breast cancer growth. PTP4A2 can regulate the invasion and migration of human lung cancer cells through ERK-dependent signaling pathway [25–28]. PTP4A2 can also regulate AKT/GSK3*β*/*β*-catenin pathway to induce EMT and promote colon cancer metastasis. PTP4A2 has been implicated in Notch1-induced and AML1-ETO-induced T cell leukemia [29, 30]. Similarly, we found that the PTP4A2 expression was significantly upregulated in hepatoma tissues, and Kaplan-Meier curves showed that the PTP4A2 overexpression from TCGA was significantly associated with shorter survival in hepatoma patients. Furthermore, we explored whether miRNA-130a-5p can be targeted by PTP4A2 in hepatoma cells. Our results demonstrated that PTP4A2 was overexpressed in hepatoma tissues. Moreover, the PTP4A2 expression was negatively related to that of miRNA-130a-5p in hepatoma tissues. Furthermore, the luciferase reporter assays revealed that miRNA-130a-5p could bind to the PTP4A2-3′UTR. The rescue experiments indicated that PTP4A2 promoted hepatoma cell proliferation and reversed the effect of miRNA-130a-5p. These findings imply that PTP4A2 is a direct target of miRNA-130a-5p.

In summary, our results showed that miRNA-130a-5p was downregulated in hepatoma tissues, and its overexpression could reduce the proliferation of hepatoma cells by targeting PTP4A2. Therefore, miRNA-130a-5p can be used as a potential biomarker for the diagnosis and prognosis of hepatoma and provided a targeted pathway for the treatment of this disease. However, we only investigated the effects of miRNA-130a-5p and PTP4A2 on hepatoma development and progression. Therefore, we need to conduct further studies to clarify the molecular mechanism underlying the effects of miRNA-130a-5p and PTP4A2, as well as to discover more therapeutic targets.

## 5. Conclusion

In conclusion, miRNA-130a-5p is downregulated in hepatoma and can worsen the prognosis of hepatoma patients. Additionally, it inhibits hepatoma cell proliferation by targeting PTP4A2. The findings provide new insights into the treatment of hepatoma.

## Figures and Tables

**Figure 1:** Downregulated expression of miRNA-130a-5p in hepatoma tissues and cell lines. (a) Expression levels of miRNA-130a-5p in 40 pairs of hepatoma and control tissues, as detected by qRT-PCR. (b) Expression levels of miRNA-130a-5p in normal LO2 cells and hepatoma cell lines. (c) Expression levels of miRNA-130a-5p in hepatoma and control tissues, as determined by GEPIA. ^∗^*P* < 0.05; ^∗∗^*P* < 0.01; ^∗∗∗^*P* < 0.001. All data are shown as mean ± SEM.

**Figure 2:** miRNA-130a-5p overexpression inhibits the proliferation of hepatoma cells. (a) HCC-LM3 cell line was transfected with LV-miRNA-130a-5p or negative control (NC). Expression levels of miRNA-130a-5p were detected by qRT-PCR. (b) Hep3B cell line was transfected with si-miRNA-130a-5p or si-NC. (c, d) CCK-8 assay data for the hepatoma cell lines with miRNA-130a-5p knockdown or overexpression. (e)–(h) Colony formation assay data for the hepatoma cell lines with miRNA-130a-5p knockdown or overexpression.

**Figure 3:** PTP4A2 is overexpressed in hepatoma tissues and associated with poor survival. (a) Venn diagram revealing 15 putative genes targeting miRNA-130a-5p based on starbase, Diana, miRDB, and miRWalk. (b) Expression levels of PTP4A2 in hepatoma tissues, as determined by qRT-PCR. (c) Spearman correlation analysis revealed the association between miRNA-130a-5p and PTP4A2 gene in 40 hepatoma specimens. (d) GEPIA database showed that PTP4A2 was increased in hepatoma tissues. (e) Kaplan-Meier curves for the survival rates of hepatoma patients with different PTP4A2 levels based on GEPIA database. (f) Dual-luciferase reporter activities of the cells transfected with WT-PTP4A2-3′UTR or MUT-PTP4A2-3′UTR as well as LV-miRNA-130a-5p, si-miRNA-130a-5p, or NC. (g) The target sequences of WT-PTP4A2-3′UTR and MUT-PTP4A2-3′UTR. (h, i) Expression levels of PTP4A2 in cells transfected with si-miRNA-130a-5p or NC and LV-miRNA-130a-5p or NC, as detected by qRT-PCR. ^∗^*P* < 0.05; ^∗∗^*P* < 0.01; ^∗∗∗^*P* < 0.001. All values are shown as mean ± SEM.

**Figure 4:** PTP4A2 overexpression reverses the effect of miRNA-130a-5p. (a) Expression levels of PTP4A2 in Hep3B cells cotransfected with PTP4A2 shRNA, miRNA-130a-5p inhibitors, and the respective controls, as determined by Western blotting. (b) Expression levels of PTP4A2 in LM3 cells cotransfected with LV-PTP4A2, LV-miRNA-130a-5p, and the respective controls, as determined by Western blotting. (c)–(f) Cell proliferation assays demonstrated that PTP4A2 promoted hepatoma cell viability and reversed the effect of miRNA-130a-5p on hepatoma cell proliferation.

**Table 1:** Correlations between miRNA-130a-5p and the clinicopathological parameters of hepatoma patients (*n* = 40, *χ*^2^ test).

Variable	MiRNA-130a-5p expression		*P* value
	High	Low	
	20	20	
Age (year)			0.097
<60	10	4	
≥60	10	16	
Gender			0.723
Female	6	5	
Male	14	15	
Tumor size			0.004^∗^
<5 cm	6	16	
≥5 cm	14	4	
TNM stage			0.011^∗^
I–II	7	16	
III–IV	13	4	
Liver cirrhosis			0.677
Yes	16	17	
No	4	3	
AFP (ng/mL)			0.157
≤200	12	17	
>200	8	3	
HBsAg			0.273
Positive	17	13	
Negative	3	7	
Edmondson grade			0.024^∗^
I–II	8	16	
III–IV	12	4	
^∗^ *P* < 0.05			

## Data Availability

The datasets generated for this study are available from the corresponding author on reasonable request.
